The article "TOX Acts an Oncological Role in Mycosis Fungoides" was retracted in 2023. Reasons: duplicate publication; signs of a paper mill; compromised peer review; concerns about the authorship.

# TOX Acts an Oncological Role in Mycosis Fungoides

**DOI:** 10.1371/journal.pone.0117479

**Published:** 2015-03-26

**Authors:** Xin Yu, Yixin Luo, Jie Liu, Yuehua Liu, Qiuning Sun

**Affiliations:** Department of Dermatology, Peking Union Medical College Hospital, Chinese Academy of Medical Sciences & Peking Union Medical College, Beijing, 100730, China; University of Medicine, Greifswald, Germany, GERMANY

## Abstract

Mycosis fungoides (MF) is a low-grade lymphoma characterized by clonal expansion of atypical CD4+ skin-homing T lymphocytes. Herein, we examined the role of thymocytes selection associated HMG-box (TOX), a gene previously found to be unregulated in MF skin biopsies, in MF pathogenesis. TOX encodes a high-mobility group family (HMG) domain DNA binding nuclear protein, which regulates the differentiation of developing T-cells. First, we confirmed that TOX expression levels in MF were increased compared with those in benign inflammatory dermatitis (BID) and normal skin. In addition, TOX level increased with the progression MF from patch stage to tumor stage. Overexpression of TOX accelerated the proliferation and migration of MF cell lines in vitro, which were blocked by AKT inhibitors. In conclusion, our study confirmed that TOX was highly expressed in MF lesions and accelerates the proliferation and migration of MF. TOX is a diagnostic marker for MF and may play a pathogenic role in disease progression.

## Introduction

Mycosis fungoides (MF) is the most common type of primary cutaneous lymphoma(PCL), a malignant disease initially affecting the skin.[1,2] MF is characterized by a clonal expansion of atypical CD4+ skin-homing T lymphocytes.[3] MF has an indolent and prolonged clinical course over years or sometimes decades, progressing from patches to more infiltrated plaques and eventually to tumors. In early stage, MF is mostly limited to skin, but in advanced cases of MF, malignant lymphocytes may disseminate to lymph nodes, peripheral blood and visceral organs. The survival rate for MF critically depends on the stages of the disease. The diagnosis of MF is mainly based on an integrated algorithm of clinical and histological criteria.[4] However, the diagnosis of early stage MF (eMF, patch and early plaque MF) is challenging even for experienced dermatologists, because of the morphologic and histological similarities of MF to benign inflammatory dermatitis (BID).[5] Quite recently, TOX was proposed as a potential molecular marker for the diagnosis of MF since its expression was higher in MF, distinguishing it from BID.[6] In addition, TOX staining was observed at a higher frequency in many different subtypes of CTCLs, including MF, Sézary Syndrome (SS), and Peripheral T-cell lymphoma, not otherwise specified (PTCL-NOS). [7] TOX was proved to be the target gene of miR-223 in CTCL.[8]

TOX (thymocyte selection associated HMG-box) encodes a high-mobility group family (HMG) domain DNA binding nuclear protein. TOX is primarily expressed in the thymus and downregulated before CD4^+^ T cells exit the thymus. TOX mRNA and proteins were poorly expressed in peripheral lymphoid tissue.[9,10] In recent years, TOX gene has been proved to be aberrant expressed in various tumors, such as lung cancer, breast cancer and leukemia.[11–14] In addition, recent studies showed that the TOX gene is highly expressed in eMF lesion in comparison to controls.[6] However, the role of TOX in malignancies has not been studied yet. The aim of this study was to further examine the role of TOX in MF. Our findings suggest that TOX plays an oncogenic role in MF, providing a possible target for the treatment of CTCL.

## Materials and Methods

### Ethics Statement

All patients or patients’ parents on behalf of the children agreed to participate in the study and gave written informed consent. Skin biopsies of MF, BID, and NS were obtained with fully informed written consent and the Clinical Research Ethics Committee of the Peking Union Medical College Hospital approval from patients undergoing biopsy in accordance with the Declaration of Helsinki Principles.

### Patients and samples

MF skin samples (patch stage, n = 21; plaque stage, n = 10; tumor stage, n = 4) were obtained from Peking Union Medical College Hospital under its approved protocols. Skin samples of BID from 10 cases each of psoriasis, chronic atopic eczema and lichen planus were selected from the tissue bank of the Peking Union Medical College Hospital. Normal skin specimens were obtained from the patients undergoing surgery at the plastic and constructive surgery department of the Peking Union Medical College Hospital. The diagnosis was based on a combination of clinical, histological, and confirmed by at least 3 dermatopathologists. Medical records were reviewed to confirm the clinical and pathological relation. MF and BID skin specimens for real-time RT-PCR and Western Blotting were obtained from patients undergoing skin biopsy at the dermatologic clinics of the Peking Union Medical College Hospital. Freshly obtained full-thickness skin samples were frozen in the liquid nitrogen until RNA or protein extraction.

### Immunohistochemistry

Formalin-fixed, paraffin-embedded sections were stained with antibodies to TOX and CD4. We used polyclonal rabbit antihuman TOX antibody (1:500dilution, Sigma, St Louis, MO, USA), followed by ABC colorimetric detection (Vector Lab, Burlingame, CA). Immunohistochemical stains for each patient were interpreted by 2 dermotopathologists. The percentage of neoplastic cells positive for TOX was scored as follows:-, no or occasional (<10% = tumor cells stained; +(10–50%) and ++(>50%) tumor cells stained.

### RNA Isolation and Quantitative Real-Time RT-PCR

The skin tissue was washed with physiologic saline and then frozen with liquid nitrogen. Total RNA was extracted using Trizol reagent (Invitrogen, Carlsbad, CA) following the instructions. Quantitative Real-Time RT-PCR was performed using the standard curve method. The sequences for primers are shown in Table 1. The relative expression of the gene of interest was assessed by the DDCt method with GAPDH as the internal control.

**Table 1:** Primer sequences for TOX, CD4 and GAPDH.

Gene	Forward Primer	Reverse Primer	Tm (°C)	Product size (bp)
TOX	TTCTCTGTGTCACCCCATGA	TCTGGCATCACAGAAATGGA	56	162
CD4	CGAAAACAGGAAAGTTGCATCA	GCCTTCTCCCGCTTCGAGAC	56	889
GAPDH	TCAACGACCACTTTGTCAAGCTCAGCT	GGTGGTCCAGGGGTCTTAC	56	116

### Protein extraction from tissues and Western blotting

The skin tissues were homogenized by mechanical disruption for 30 min at 4°C and then incubated in lysis buffer (50 mmol ⁄ L Tris, pH 7.5, 150 mmol⁄L NaCl, 1 mmol⁄ L EDTA, 1% Triton X-100, 1% sodium deoxycholate, 0.1% SDS, 1 lmol ⁄ L phenylmethylsulfonyl fluoride, 5 lg ⁄ ml aprotinin). After centrifugation at 12 000 rpm for 20 min at 4°C, the supernatant was obtained. Total protein from the supernatant was quantified using the Bradford assay (Sigma, St Louis, MO, USA). After being subjected to SDS–PAGE, protein extracts were transferred to a PVDF membrane (Millipore, MA). They were then incubated with primary antibodies against the following protein: TOX (dilutions 1:500, Sigma, St Louis, MO, USA), p-AKT (dilutions 1:2,000, Abcam)and GAPDH (dilutions 1:2,000, Abcam). Protein bands were then visualized with HRP-conjugated secondary antibody (1: 1,000 dilution, Abcam) and ECL kit (Millipore).

### Cell Culture and transfection

Myla (MF cell line) were obtained from European Collection of Cell Cultures (ECACC). Cells were cultured in serum-free RPMI1640 (Millipore, Billerica, MA). TOX vector and siRNA were designed and synthesized by GenePharma (Shanghai, China) and were performed with Lipofectamine 2000 (Dharmacon, TX, USA) according to the manufacturer’s instructions. Transfection complexes were prepared according to the manufacturer’s instructions.

### Cell proliferation assay

Cells were incubated in 10% CCK-8 (Dojindo; Kumamoto, Japan) that was diluted in normal culture medium at 37°C until the visual color conversion occurred. Proliferation rates were determined at 0, 24, 48 and 72 hours after cell transfection.

### Cell migration and invasion assay

In order to conduct the Transwell migration assays, 5 × 10^4^ cells were plated in the upper chamber of the insert with 8-μm pore size filters (BD Bioscience). For invasion assays, 1×10^5^ cells were added into the top chamber of the insert filter, which was precoated with Matrigel (BD Bioscience). In both of the migration and invasion assays, cells were plated in medium without serum. The lower chamber medium contained 10% FBS as a chemo attractant. The cells were then cultured for 48 h. MF cells that migrated to the underside of the membrane were fixed with methanol and stained with Giemsa. Then they were imaged and counted.

### Statistical analysis

Statistical analysis was performed using SPSS ver. 18.0 software. P < 0.05 was considered statistically significant. The results of average OD and relative grey scale were expressed as mean ± standard deviation (mean ± SD). Statistical analysis was performed using Student’s t-test.

## Results

### Expression of TOX in MF by immunohistochemistry, Real-Time RT-PCR and Western Blotting

In 32 of 35 (91%) biopsies, more than 10% of the neoplastic T cells showed clear nuclear staining for TOX, whereas only 6 of 30 (20%) BID specimen showed over 10% positive staining (Table 2). There was a significant difference between MF and BID or healthy skin (Table 3, P<0.0001, Chi-square test). By comparison, the number of cells expressing TOX increased with the lymphoma progression from patch stage to tumor stage (Fig. 1). In the eMF skin biopsies, TOX labeled the MF cells in Pautrier’microabscess (Fig. 2). Taken together, our results demonstrated a significant difference in the expression TOX between MF and BID. In addition, TOX expression was increased with the progression MF from patch stage to tumor stage (Table 3). Consistent with the results of the immunohistochemical staining, the mRNA levels and protein levels of TOX in MF were also higher compared with that in BID and NS samples (Fig. 3 and Fig. 4).

**Fig 1:** Representative immunohistochemical staining of TOX in different stages of MF lesions. (A) Patch stage MF. Only a few infiltrating MF cells were positive for TOX while the majority of lymphocytes stained negative. (B) Plaque stage MF. Atypical infiltrating lymphocytes in the dermis were positive for TOX. (C) Tumor stage MF. The majority of infiltrating lymphocyteswere stained positive.

**Fig 2:** Representative immunohistochemical staining for TOX and CD4 in a patch stage MF lesion. Bright focal nuclei staining on lymphoid cells were considered to be positive. The arrow indicates the epidermotropic MF cells in a Pautrier’s microabscess and papillary dermal MF cells staining positive with TOX and CD4.

**Fig 3:** The TOX expression in MF lesion by real-time RT PCR. (A) TOX mRNAs in MF、BID and NS. (B) CD4 mRNAs in MF、BID and NS. RT-PCR analysis was performed in triplicate and the expression levels of TOX and CD4 mRNAs were normalized to GAPDH mRNAs. Error bars represent as SD.

**Fig 4:** The TOX expression in MF lesion by Western blot analysis. (A) CD4 protein expression in MF、BID and NS. (B) TOX protein expression in MF、BID and NS.The signal in each lane was quantified using Image J software and the ratio of TOX and CD4 to GAPDH were determined. Error bars represent SD. MF mycosis fungoides, BID Benign inflammatory diseases, NS Normal skin

**Table 2:** TOX expression in MF and comparison group.

Tissue types	Total no.	Pos no. (%)	X2	p
MF	35	32(91%)		
BID	30	6(20%)		<0.0001
NS	30	0(0%)		<0.0001

All p values were compared to MF.

MF mycosis fungoides, BID Benign inflammatory diseases,NSNormal skin, Pos no. positive numbers

**Table 3:** TOX expression in different stage of mycosis fungoides.

Diagnosis	Percentage of nuclei expressing TOX		
	-	+	++
Patch stage (n = 21)	2 (10%)	15 (71%)	4(19%)
Plaque stage (n = 10)	1(10%)	2(20%)	7 (70%)
Tumor stage (n = 4)	0(0%)	0(0%)	4 (100%)
BID (n = 30)	24 (80%)	6 (20%)	0 (0%)
Normal Skin (n = 30)	30(100%)	0	0

### TOX accelerates the MyLa cell proliferation

Western blot assays showed that TOX vector enhanced the expression of TOX (Fig. 5A). CCK8 assays showed that TOX increased MF cell proliferation compared with either the control vector-transfected cells or the untreated cells (Fig. 5B). Moreover, our result has shown that overexpression of TOX can enhance the cell cycle progression (Fig. 5C).The proliferative effect of TOX was further confirmed by real-time PCR and Western blot of Ki-67.As is shown in Fig. 5D and E, there was a significant increase in the protein and mRNA of Ki-67 in the group transfected with TOX vector as compared with the control group or untreated group.

**Fig 5:** TOX accelerates the MyLa cell proliferation. (A) Western blot analysis showed that TOX vector could enhance the expression of TOX. The expression of TOX was normalized to GAPDH. (B)CCK8 assays have showed that overexpression of TOX increased the Myla cell proliferation compared with either the control vector-transfected cells or the untreated cells. (C)The effect of TOX on cell cycle progression of the Myla cell after 48-h incubation was detected by flow cytometry analysis. (D) TOX promoted Ki-67 mRNA expression. The Myla cells were transfected with TOX vector, controlornot transfected. Ki-67were detected by real-time PCR.(E)TOXpromotedKi-67protein expression. The Myla cells were transfected with TOX vector, controlornot transfected. Ki-67was detected by western blot.The expression of ki-67 was normalized to GAPDH. Values are presented as mean±SD. As compared with control, ** p<0.01, *p<0.05, and ***p<0.001

### TOX accelerates the MyLa cell migration and invasion

We performed migration and invasion assay to investigate the effects of TOX on the migratory and invasive behaviors of MyLa cells in vitro. Cells in the TOX vector group exhibited increased migration and invasion as compared with cells in the control group or untreated group respectively (Fig. 6A and B).

**Fig 6:** TOX accelerates the MyLa cell migration and invasion. (A) Migration assays of the Myla cells after treatment with TOX vector, control or not transfected; the relative ratio of migratory cells per field is shown on the right.(B) Invasion analysis of the Myla cells after treatment with TOX vector, control or not transfected; the relative ratio of invasive cells per field is shown on the right, ***p<0.001.

### TOX stimulatesMF cell proliferation and invasion through AKT phosphorylation

Western blot assays showed that overexpression of TOX stimulated AKT phosphorylation (Fig. 7A). In addition, this proliferative effect was inhibited by LY294002, an AKT inhibitor (Fig. 7B). Moreover, the changes in invasion after TOX overexpression was largely blocked by LY294002 (Fig. 7C). Thus, overexpression of TOX results in LY294002-sensitive activation of AKT, a major cell survival factor.

**Fig 7:** TOX stimulated MF cell proliferation and invasion through AKT phosphorylation. (A) Western blot assays showed that LY294002 can inhibited AKT phosphorylation. The expression of p-AKT was normalized to GAPDH. (B) Western blot assays showed that overexpression of TOX stimulated AKT phosphorylation. The expression of p-AKT was normalized to GAPDH. (C) The proliferative role of TOX overexpression was largely blocked by LY294002, an AKT inhibitor, in MyLa cells were transfected with TOX vector, control or not transfected or TOX vector and LY294002. (D) The invasive role of TOX overexpression was largely blocked by LY294002, an AKT inhibitor, in MyLa cells were transfected with TOX vector, control or not transfected or TOX vector and LY294002. ** p<0.01, *p<0.05, and ***p<0.001.

## Discussion

In the present study, TOX was overexpressed in all stages of MF and TOX expression was increased with the progression MF from patch stage to tumor stage, suggesting a correlation of TOX with the progression of tumors. More importantly, we demonstrated that TOX promoted MF cell proliferation and migration, through AKT pathway. As far as we know this is the first study analyzing the roles of TOX in MF.

TOX contains a DNA- binding domain, which allows it to regulate transcription by modifying local chromatin structure and modulating the formation of multi-protein complexes[10]. TOX plays a critical role in T-cell development although the exact function remains unclear and the circumstances when TOX is expressed remain unclear. TOX is highly expressed in the thymus and in developing T cells, but after exiting thymus and entering the peripheral tissue, mature CD4+ T cells never again expressed TOX to a significant level.[15,16] Under normal condition, TOX gene is mainly expressed in the thymus followed by the liver and brain; it is poorly expressed or absent in normal skin.[17] Since TOX demonstrated highly specific staining of MF cells in the early epidermotropic cells in Pautrier’s microabscesses, we conclude that TOX is primarily derived from the malignant clone of MF cells, different from the normal immune response in tumor immunity. However, whether the high expression of TOX was involved in the appropriate control of the immune response in MF remains unclear. Further investigations are needed.

Accumulating evidence has showed that TOX was deregulated in various malignancies, including breast cancer, lung cancer[11,12]. As far as we know, this is the first report describing the function of TOX in tumor, as well as the MF.[7,18] Zhang et al. first suggested TOX as the molecular markers for histological diagnosis of eMF, since they found that TOX was overexpressed in eMF compared with BID[6]. Later Huang et al. confirmed the hypothesis in a full spectrum of MF skin biopsies [18]. Consistent with their findings, we also found that TOX was overexpressed in MF compared with BID, suggesting its potential role as molecular diagnostic markers for MF. In addition, we found that TOX expression was increased with the progression MF from patch stage to tumor stage. However, the functional significance of TOX expression and its role in MF cell proliferation and migration has never been explored previously. In vitro experiment has shown that TOX promoted Myla cell proliferation and migration. In addition, knockdown of TOX expression by siRNA decreased Myla cell proliferation and migration. Those results indicate that TOX might play an oncogenic role in MF by promoting cell proliferation and migration. Although in vitro data supports that overexpression of TOX can promote Myla cell proliferation and migration, further experiments are needed to measure the functional role of TOX in the nude mice. The phosphoinositide 3-kinase (PI3K)/AKT signaling is one of the most critical regulatory pathways in cancer[19]. Since aberrant activation of AKT has been reported in CTCL[20–22], we examined whether it is involved in TOX. In our study, overexpression of TOX stimulated AKT phosphorylation and AKT inhibitor inhibited the proliferative effect induced by TOX. Thus we concluded that TOX might promote cell proliferation and spread through activating AKT and the PI3K/AKT signal pathway.

In conclusion, our results demonstrated the overexpression of TOX in MF skin lesions and its relation with the progression of MF. We also indicated that TOX promoted MF cells proliferation and migration through activating AKT pathway. Since the pathogenesis of MF remains largely unknown. The investigation of the role of TOX and the related mechanism may provide some insights into the understanding pathogenesis of MF. In addition, TOX may be a potent target for the development of molecular markers and therapeutic strategies for patients with MF.
